# CY-09 Inhibits NLRP3 Inflammasome Activation to Relieve Pain via TRPA1

**DOI:** 10.1155/2021/9806690

**Published:** 2021-08-14

**Authors:** Youjia Fan, Gaici Xue, Qianbo Chen, Ye Lu, Rong Dong, Hongbin Yuan

**Affiliations:** ^1^Department of Anesthesiology, Changzheng Hospital, Second Military Medical University, Shanghai 200003, China; ^2^Department of Neurosurgery, Southern Theater Command of the People's Liberation Army, Shanghai 510010, China; ^3^Department of Anesthesiology, The Third Affiliated Hospital of Naval Military Medical University, Shanghai 200438, China; ^4^Department of Anesthesiology, Ruijin Hospital, Shanghai Jiao Tong University, Shanghai 200000, China

## Abstract

Peripheral tissue damage leads to inflammatory pain, and inflammatory cytokine releasing is the key factor for inducing the sensitization of nociceptors. As a calcium ion channel, TRPA1 plays an important role in pain and inflammation, thus becoming a new type of anti-inflammatory and analgesic target. However, there is no consensus on the role of this channel in mechanical hyperalgesia caused by inflammation. Here, we aim to explore the role and underlying mechanism of the inflammasome inhibitor CY-09 in two classic inflammatory pain models. We evaluated pain behavior on animal models, cytokine levels, intracellular Ca^2+^ levels, transient TRPA1 expression, NF-*κ*B transcription, and NLPR3 inflammasome activation. Consistently, CY-09 reduced the production of inflammatory cytokines, intracellular Ca^2+^ levels, and the activation of TRPA1 by inhibiting the activation of inflammasomes, thereby reducing the proinflammatory polarization of macrophages and alleviating animal pain and injury. Importantly, AITC (TRPA1 agonist) significantly reversed the analgesic effect of CY-09, indicating that TRPA1 was involved in the analgesic effect of CY-09. Our findings indicate that CY-09 relieves inflammation and pain via inhibiting TRPA1-mediated activation of NLRP3 inflammasomes. Thus, NLRP3 inflammasome may be a potential therapeutic target for pain treatment and CY-09 may be a pharmacological agent to relieve inflammatory pain, which needs further research.

## 1. Introduction

Pain is an unpleasant emotion and sensory experience resulting from tissue damage. Currently, there are three modes of pain: pathological pain, nociceptive pain, and inflammatory pain [1, 2]. Inflammatory pain is mainly caused by intracellular ion accumulation and inflammatory mediator secretion, such as prostaglandin, serotonin, and bradykinin. Inflammatory pain is accompanied by many diseases, including diabetes, cancer, infection, autoimmune disease, chemotherapy, and trauma. Furthermore, most patients are always with mental symptoms, such as anxiety, depression, and insomnia, which seriously affect the quality of life [3–6]. Pain and depression aggravate each other. Some inflammation, such as arthritis, can cause the central nervous system to be stressed too much, which leads to central sensitivity, and then causes chronic pain and emotional distress to worsen [7]. People suffering from pain and inflammation are more depressed, leading to increased suicide rates and burden social and public security. Therefore, finding specific molecular targets and developing potent, safe, and low-tolerated analgesics become a hotspot in pain treatment research.

Transient receptor potential ankyrin 1 (TRPA1) is a calcium-permeable cation channel and belongs to the TRP channel superfamily [8]. TRPA1 is widely expressed in the nervous system, digestive system, and respiratory system, involving the regulation of nerve excitability and the function of various organs. TRPA1 channel plays an important role in pain and inflammation, becoming a novel type of anti-inflammatory and analgesic target [9, 10]. Different agonists can regulate the physiological functions of the body or induce pathological damage by upregulating the function of TRPA1 channels. In the absence of TRPA1, heat hyperalgesia disappears after administration of complete Freund's adjuvant (CFA) or carrageenan in mice; TRPA1 knockout mice have limited histological changes in the model [11–13].

Many researchers have discovered that IL-1*β* and IL-18 secrete during the process of inflammatory pain and promote NLRP3 inflammasome assembling [14, 15]. Activated NLRP3 and ASC form a scaffold to stimulate procaspase-1 and promote the hydrolysis of pro-IL-1*β* and pro-IL-18. To date, several studies demonstrate that NLRP3 inflammasome acts as a “relay station” in the pain process [16]. For instance, in the CCI rat pain model, morphine treatment causes p38 phosphorylation and NLRP3 activation resulting in continuous nociceptive stimulation [17]. Electroacupuncture (EA) could inhibit the activation of NLRP3 inflammasome relieving inflammatory pain [18]. Although some studies have reported NLRP3 inflammasomes involve inflammatory pain, the mechanism of its downstream molecules and whether its inhibitors can be used as pain treatment remain unclear.

CY-09 is an NLRP3 inhibitor, by binding to its NACHT domain to inhibit ATPase activity [19]. CY-09 effectively inhibits IL-1*β* production and the influx of neutrophils in the monosodium urate (MSU) injection-induced gout model, suggesting CY-09 plays a vital role in blocking NLRP3 inflammasome activation *in vivo.* CY-09 treatment can also suppress noncanonical NLRP3 activation induced by cytoplasmic LPS in BMDM [19]. Though CY-09 has been used in some pain models, the mechanism remains unclear.

In our study, based on the hypothesis that CY-09 can inhibit NLRP3 inflammasome formation and reduce TRPA1 channel activation to alleviate inflammatory pain, we find that inhibition of TRPA1-mediated activation of NLRP3 inflammasomes is related to the analgesic effect of CY-09 on inflammatory pain.

## 2. Materials and Methods

### 2.1. Animals

C57/BL6 mice (6-8 weeks, 22 g) were purchased from the Second Military Medical University, Center of Laboratory Animals and acclimated for 1 week before the experiment (production license no. SCXK (hu)2012-0003). The Animal Care Facility was approved by the Animal Care and Use Committee of Changzheng Hospital and followed the guide.

### 2.2. Thermal Withdrawal Latency Test

The mice were placed on a hot plate, and the heat stimulated the mouse's feet to produce a pain response. The time for the mice to lick feet was used as an indicator of pain response and to determine whether the drug had an analgesic effect. We first chose mice with pain response within the 30 s as normal, placed the mouse in a 55 ± 0.5°C hot plate apparatus, and used the mouse's hindfoot as an observation index to determine the pain threshold of the mouse. The measurement was performed twice every 5 minutes.

### 2.3. Paw Licking Time Test

Mice were injected with LPS or formalin on their pelma and then treated CY-09 through intragastric administration. Paw licking time was measured in a blinded fashion after the LPS or formalin challenge. Each group of mice was observed and counted the licking time within 60 minutes.

### 2.4. Real-Time Quantitative PCR

The RNA extraction kit (Qiagen, Germany) was introduced to isolate total RNA from feet tissue. After reverse transcription array, real-time quantitative PCR was performed using SYBR Green PCR master mix and analyzed with a Light Cycler 480 (Roche, Germany). The expression was tested using specific primers. The IL-6 sense primer was 5′-TAAGCCTCCGACTTGTGAAGTGGT-3′, and the antisense primer was 5′-ATCCAGTTGCCTTCTTGGGACTGA-3′; the IL-1*β* sense primer was 5′-CAGGCAGGCAGTATCACTCA-3′, and the antisense primer was 5′-AGCTCATATGGGTCCGACAG-3′; the TNF-*α* sense primer was 5′-CATCTTCTCAAAATTCGAGTGACAA-3′, and the antisense primer was 5′-TGGGAGTAGACAAGGTACAACCC-3′; the NLRP3 sense primer was 5′-ATGCTGCTTCGACATCTCCT-3′, and the antisense primer was 5′-AACCAATGCGAGATCCTGAC-3′; the caspase-1 sense primer was 5′-CACAGCTCTGGAGATGGTGA-3′, and the antisense primer was 5′-TCTTTCAAGCTTGGGCACTT-3′; the NF-*κ*B sense primer was 5′-CTCCCTGACAAGCCTGCTAC-3′, and the antisense primer was 5′-TCTTCCTTCAGCGTCTGGAT-3′; the TRPA1 sense primer was 5′-CTACTGGCTTTTGGCCTCAG-3′, and the antisense primer was 5′-CCAAAGGTCAGGACTGGGTA-3′; the GAPDH sense primer was 5′-CCGCATCTTCTTGTGCAGT-3′, and the antisense primer was 5′-GGCAACAATCTCCACTTTGC-3′.

### 2.5. Ca^2+^ Concentration Detection

The intracellular Ca^2+^ concentrations in the homogenized and centrifuged tissue samples were determined using the BioVision kit. Then, the absorbance was measured at 575 nm through a microplate reader.

### 2.6. Western Blotting

Tissues were collected and lysed with RIPA. After protein concentration detection, protein samples were loaded and membranes were incubated with primary antibodies TRPA1 (PA1-29421, Invitrogen) and GAPDH (ab181602, Abcam).

### 2.7. Flow Cytometry

Mouse foot tissues were harvested, minced into small pieces, and then digested with collagenase II and dispase II (Sigma-Aldrich, MO, USA) in PBS for 30 min at 37°C. The cell suspension was filtered, centrifuged, resuspended, and blocked with a CD16/32 antibody. Then, the cells were stained with primary antibodies in FACS buffer for 30 min at 4°C in the dark. Flow cytometry analysis was performed on a BD FACS Calibur using Diva 6 Software (BD Biosciences, San Jose, CA, USA). The results were analyzed using FlowJo Software V10.2 (TreeStar, OR, USA).

### 2.8. Statistical Analysis

Data were analyzed using GraphPad Prism 8.0. All data were presented as means ± SEM. All experiments were repeated three times. A comparison of groups was performed using an unpaired Student's *t*-test. ^∗^*P* < 0.05, ^∗∗^*P* < 0.01, and ^∗∗∗^*P* < 0.001 indicated statistical significance.

## 3. Results

### 3.1. CY-09 Relieves Inflammatory Pain and Reduces Cytokine Production in Mice Induced by LPS or Formalin

The CY-09-pretreated mice were treated with LPS or formalin, and two different models were used to induce inflammatory pain. Compared with formalin-induced inflammation, LPS was slower and lasted longer. The degree of pain was evaluated by hot plate time and foot licking time. After injection, mouse pain behavior was obvious and the foot tissue became swelling. 5 mg/kg of CY-09 obviously inhibited thermal hyperalgesia induced by LPS at 5 h (Figure 1(a)) and formalin 1 h (Figure 1(b)), respectively. Additionally, CY-09 significantly suppressed pain, and its analgesic behavior always existed within 60 minutes.

White blood cells enriched during inflammatory pain occur and repair the damaged tissue. The production of inflammatory cytokines is an important indicator in the process of inflammatory pain. We further evaluated the expression of inflammatory factors in the plantar tissue through RT-qPCR. We first detected IL-6 and TNF-*α*, two indicators in the process of acute inflammation. Data suggested that CY-09 could relieve inflammatory cytokine release (Figures 1(c) and 1(d)). Then, we tested the IL-1*β* expression level. The results showed that the extracellular secretion level of IL-1*β* was upregulated in the two models induced by LPS and formalin, but then, it was inhibited by CY-09 (Figures 1(c) and 1(d)). Thus, CY-09 relieved pain by reducing the level of inflammation.

### 3.2. CY-09 Suppresses NF-*κ*B Transcription and NLPR3 Inflammasome Activation and Reduces Macrophage M1 Polarization

To explore the underlying mechanisms of the CY-09 antinociceptive effect, we examined the activation of the classic inflammation pathway NF-*κ*B and inflammasome pathway. RT-PCR data indicated that CY-09 reduced NLPR3, ASC, and caspase-1 expression in LPS or formalin-induced mice (Figures 2(a) and 2(b)). In addition, CY-09 significantly suppressed nuclear NF-*κ*B (p65) transcription (Figures 2(a) and 2(b)). Next, we investigated macrophages recruited during the activation of NLRP3 in foot tissues. We used CD45 and F4/80 two indicators to distinguish the total amount of white blood cells and defining iNOS+ as M1 polarization and CD206+ as M2 polarization. Compared with the nontreatment group, the percentage of M1 was decreased and the M2 marker was increased (Figure 2(c)). These findings suggested that CY-09 application reduced macrophage M1 polarization and weakened the secretion of proinflammatory factors.

### 3.3. CY-09 Inhibits TRPA1 Expression *In Vivo*

It is reported that the TRPA1 channel is involved in the activation of the NLPR3 inflammasome, and we hypothesize that CY-09 could regulate TRPA1 expression. After LPS administration, the expression of TRPA1 in the footpad tissues was significantly upregulated. However, CY-09 significantly reduced TRPA1 expression (Figures 3(a) and 3(b)). TRPA1 is a calcium ion channel. We further evaluated the calcium ion level in the tissue. Compared with the single LPS injection group, the CY-09 treatment significantly reduced the intracellular Ca^2+^ concentration (Figure 3(c)). In the formalin-treated model, we also found similar results as the LPS-treated model (Figures 3(d)–3(f)).

### 3.4. TRPA1 Is Involved in the Antinociceptive Effect of CY-09

Since TRPA1 might be the main cause of intracellular calcium elevation, AITC (TRPA1 agonist) and inhibitor HC030031 were used to further evaluate. AITC decreased the inhibitory effect of CY-09 in LPS-induced thermal hyperalgesia and licking times, although mice treated with AITC alone had no obvious effect (Figures 4(a)–4(c)). As shown in Figure 5, AITC as a specific agonist significantly enhanced the expression of TRPA1(Figure 5(b)). In addition, AITC reversed the activity of CY-09 in the inhibitory intracellular Ca^2+^ levels and IL-1*β* and TNF-*α* production (Figures 5(a) and 5(c)). Finally, NLPR3 inflammasome activation was also evaluated. The results showed that AITC could reverse the reduction of cytoplasmic and NLPR3 activation induced by CY-09 (Figure 5(d)).

## 4. Discussion

Direct injection of formalin or LPS into the paw of the mouse is a common model of inflammatory pain. The formalin model mainly represents the spontaneous pain behavior and hypersensitivity of mechanical and thermal stimulation [20]. LPS, as a major factor of gram-negative bacteria, binds to Toll receptors and triggers an intracellular signal cascade and subsequently produces inflammatory cytokines, causing neutrophil and macrophage recruitment [14, 21]. In this study, we used two different animal models. It was found that there were typical features of inflammatory pain in both models, including hyperalgesia, paw edema, and macrophage infiltration. We found that NF-*κ*B transcription had a positive regulatory role in the activation of NLRP3/ASC/procaspase-1/pro-IL-1*β*. Under stimulation, LPS or formalin enhanced NF-*κ*B (p65) phosphorylation and promoted the assembly of NLRP3/ASC/procaspase-1 inflammasomes, resulting in the cleavage of caspase-1 and IL-1*β* secretion. IL-1*β* further maturation and secretion polarized macrophages to proinflammatory mode M1.

More and more evidence shows that NLRP3 inflammasome is involved in inflammatory pain. NLRP3 inflammasome activation, ASC rapidly distributes from the nucleus to the cytoplasm and participates in the activation of caspase-1 precursors [15, 22, 23]. Regardless of the CCI, SCI, or SNL-induced mouse model, NLRP3, caspase-1, and ASC expressions were not only increased in peripheral dorsal root ganglia and neurons but also expressed in microglia and astrocytes [24, 25]. However, there are also conflicting results. Research indicates that NLRP3 inflammasome and IL-1*β* do not participate in the occurrence of the pain model [26]. We speculate that NLRP3 inflammasomes may play different roles in individual pain models and need further confirmation. Since NLRP3 plays a key role in pain, NLRP3 may be a potential therapeutic target. Therefore, it is particularly important to confirm that NLRP3 activates mechanisms and functions in different pain models. In our work, in addition to the activation of inflammasomes, the promotion of the secretion of proinflammatory factors, and the activation of macrophages, we also find that the intracellular Ca^2+^ concentration increases in the tissues.

The elevation of intracellular Ca^2+^ levels is due to the release of Ca^2+^ storage from the endoplasmic reticulum [27]. We focus on a calcium channel TRPA1. TRPA1 is a Ca^2+^ permeable cation channel. As a nociceptor, it has been considered an important target in pain treatment. Studies have found that the mutation N855S located in the transmembrane structure of TRPA1 S4 could cause familial pain syndrome, which is the first pain-related ion channel disease [28]. A variety of exogenous TRPA1 agonists can induce the body's neurotransmitter release, inflammation, and pain, such as AITC, formalin, and cinnamaldehyde. Endogenous TRPA1 agonists can also induce calcium influx and pain response in DRG neurons in a dose-dependent manner [8, 29, 30]. Our results indicate that the activation of NLRP3 inflammasomes induced by LPS is related to the increased expression of TRPA1, and TRPA1 may be the target of CY-09, indicating that TRPA1-mediated NLRP3 inflammasomes may be involved in the activation of CY-09 analgesic effect on inflammatory pain.

As an inhibitor of inflammasomes, CY-09 is reported to have analgesic activity and resist inflammatory pain [19]. It is worth noting that CY-09 could relieve inflammatory hyperalgesia caused by LPS or formalin. CY-09 also showed the ability to inhibit the activation of NLRP3 inflammasomes and recruited macrophages. In addition, the elimination effect of AITC (a special TRPA1 agonist) on CY-09 further confirms that TRPA1 is involved in inflammatory pain. In the presence of TRPA1 agonists, the inhibitory effect of CY-09 treatment on NF-*κ*B (p65) transcription cannot be reversed, indicating that other signal transduction pathways or mechanisms may be involved in the analgesic process of CY-09. However, the upstream and downstream relationships between the two TRPA1 and CY-09 are still mutual feedback and need to be further explored.

Taken together, our results reveal CY-09 relieves inflammatory pain in the mouse model, partially relating to the regulation of NF-*κ*B transcription, NLRP3 inflammasome formation, and TRPA1/Ca^2+^ mobilization. Thus, NLRP3 inflammasome may be a potential therapeutic target for pain treatment and CY-09 may be an analgesic candidate, deserving further research. This study provides an important experimental basis for studying whether NLRP3 is a potential therapeutic target for pain treatment and whether CY-09 can be used as a pharmacological drug to relieve inflammatory pain.

## Figures and Tables

**Figure 1:** CY-09 relieves inflammatory pain and inflammatory cytokine production in mice. (a, b) Effects of CY-09 on LPS or formalin-induced thermal hyperalgesia and licking time in mice with inflammatory pain. Mock (saline) or CY-09 was i.p. injected into mice (*n* = 8 per group). 2 h after the last injection, LPS (10 ng/*μ*L) was used via i.p. injection. After 5 h, mice were sacrificed by cervical dislocation and samples were collected. Thermal hyperalgesia was evaluated by the time course of the paw withdrawal latency at the indicated time points after injection using a hot plate apparatus. Licking time of each group of mice was observed and counted within 60 minutes. (c, d) Effect of CY-09 on LPS or formalin-induced inflammatory responses. Levels of IL-6, TNF-*α*, and IL-1*β* in footpad tissues were assessed by RT-PCR. ^∗^*P* < 0.05, ^∗∗^*P* < 0.01, and ^∗∗∗^*P* < 0.001. Data showed mean ± SEM.

**Figure 2:** CY-09 reduces NLPR3 inflammasome activation and promotes macrophage M2 polarization. (a, b) Effects of CY-09 on NF-*κ*B transcription and NLPR3 pathway activation. (c) Flow cytometry analysis of macrophage polarization of footpad skin. ^∗^*P* < 0.05, ^∗∗^*P* < 0.01, and ^∗∗∗^*P* < 0.001. Data showed mean ± SEM.

**Figure 3:** CY-09 inhibits TRPA1 expression in mice with inflammatory pain. (a, b) mRNA and protein levels of TRPA1 expression on the LPS-induced inflammatory model. (c) Effects of CY-09 on intracellular Ca^2+^ concentration on the LPS-induced inflammatory model. (d, e) mRNA and protein levels of TRPA1 expression on the formalin-induced inflammatory model. (f) Effects of CY-09 on intracellular Ca^2+^ concentration on the formalin-induced inflammatory model. ^∗^*P* < 0.05, ^∗∗^*P* < 0.01, and ^∗∗∗^*P* < 0.001. Data showed mean ± SEM.

**Figure 4:** Effect of TRPA1 agonists in mice with inflammatory pain. (a) Thermal hyperalgesia was evaluated by the time course of the paw withdrawal latency at the indicated time points after LPS injection using a hot plate apparatus. Mock (saline) or CY-09 was i.p. injected into mice (*n* = 8 per group). Simultaneously, AITC (TRPA1 agonists, 0.05 mg/kg) was applied via s.c. injection and two hours after the last injection, mice were subjected to LPS (10 ng/*μ*L) via i.pl. injection. (b, c) Licking time was measured and analyzed within 60 min. ^∗^*P* < 0.05, ^∗∗^*P* < 0.01, and ^∗∗∗^*P* < 0.001. Data showed mean ± SEM.

**Figure 5:** Effects of AITC (TRPA1 agonists) on cytokine production, intracellular Ca^2+^ concentration, and NLRP3 activity. (a, b) Effects of AITC on Ca^2+^ concentration and the expression of TRPA1. Mice were treated with AITC (TRPA1 agonists) as described in Figure 4. (c) Intracellular IL-6, TNF-*α*, and IL-1*β* expression level in different groups was detected and statistically analyzed. (d) The expression of NLRP3, ASC, and caspase-1 in footpad tissues of different groups was measured and analyzed. ^∗^*P* < 0.05, ^∗∗^*P* < 0.01, and ^∗∗∗^*P* < 0.001. Data showed mean ± SEM.

## Data Availability

The data that support the findings of this study are available on request from the corresponding author.
